# A wireless sensor network for coal mine safety powered by modified localization algorithm

**DOI:** 10.1016/j.heliyon.2024.e41262

**Published:** 2024-12-24

**Authors:** Hafiz Zameer ul Hassan, Anyi Wang, Ghulam Mohi-ud-din

**Affiliations:** a College of Communication and Information Engineering, Xi'an University of Science and Technology, Xi'an, 710054, China; b Department of Computer Engineering – University of Florida, Gainesville, FL, USA

**Keywords:** Coal mining industry, Modified precise, DV (Distance Vector)-Hop localization algorithm, Safety parameters, Safety alert, MATLAB

## Abstract

Coal mining industry is one of the main source for economy of every nations, whereas safety in the underground coal mining area is still doubtful. According to some reports, there is heavy loss of life and money due to the occasional accidents in the coal mining area. Some existing researchers has been addressed this issue and approached their method. But the limitations are the communication range between the anchor nodes are weak because of its complex infrastructure. In coal mines, gas leaks pose a serious safety risk, often leading to explosions or toxic exposure. Temperature control is difficult due to fluctuating underground conditions, potentially causing heat stress or equipment malfunction. Real-time worker tracking is challenging in these environments, making it harder to monitor safety and respond swiftly to emergencies. To overcome the challenges, the proposed research uses modified precise DV (Distance Vector)-Hop localization algorithm. The data is collected from the nodes and it will generate as anchor nodes and sensor nodes. The proposed research includes some parameters to analyze the abnormal environment characteristics such as network parameters, proposed localization algorithm parameters, simulation parameters, safety monitoring parameters. These parameters helps to send the safety alert to the ground center in case of any emergency such as high temperature, gas leakage, changes in air humidity. The proposed model has the ability to detect all the sensor nodes within the threshold value as well as outside the threshold value. This shows that the proposed model communication range and it accuracy is higher than the existing research. The MATLAB simulation tool is used to enhance the localization of the proposed algorithm where, it is compare the traditional DV-Hop localization algorithm. The proposed algorithm attain high performance accuracy than existing method. The efficiency of the proposed modified precise DV-Hop localization algorithm is evaluated by the simulation outcomes.

## 1 Introduction

The essential parameters in mining are worker's health and surveillance of the mining environment. While working in mining there are some unavoidable issues such as the number of people are engaged directly, the hazardous nature of mining operations, the high operational cost and investment of mining activities, the uncertainty of different mining units [1]. In the mining industry the fundamental concerns are the health issues relevant to the activities of the mine workers and occupational hazards. Due to fresh air access and adequate light, it is obvious that the safety in underground mines should be high than open pit mines [2]. The underground mines are more accident zone regarding the geology complexity, direct influence on the stress distribution type and their present continuities structure [3]. In underground mines, the existing dangers and unexpected accidents could reflect dangerous and stressful working environment and the financial and life threats are executed by the operational facilities [4]. Due to the environment developing from inadequate light, area constraints, geology complexities, environmental pollutants, etc. the working hazards in underground mines need particular attention to all mentioned triggering safety factors. Because of its bothersome ergonomy, weight and heat the workers incline to keep away some safety equipment [5]. The coal mining technology has made great contributions and full progress in meet out the national energy demand in recent years. Particularly, the method with backward production capacity is gradually replaced by the intelligent coal mining technology [6]. Conversely, in the realm of intelligent coal mine one of the research hotspot is the effective communication problem due to its deep underground [7]. Therefore, the conventional coal business is likely to elevate to the smart coal manufacturing. In the industry the other conditions to make sure the high quality and effective expansion of the prominent initiatives by necessarily make the advancement in 5G sensor networks technology [8]

Including the specific technical challenges, the quarries and mines are dynamically keep developing. Especially in underground settings, these surroundings are still dangerous for workers, even with the technological advancement [10]. Additionally, narrow working area, high temperatures, low visibility, humidity and gas concentration are the common hazards [11]. It is important to determine where the miners are in order to rescue them in case of an accident. The power cut is expected to happen when the flood or root collapse incident occurs [12]. During this period, the communication in the underground coal mining is very significant, but the traditional sensors failed to transfer the information because it not always straightforward [13]. To overcome this issue by the most popular means of achieving the objective and potential WSN (Wireless sensor network). In most cases, they emphasis a low-cost alternative, incredibly flexible and they do not need any wiring structures [14]. Through the use of Ultra Wide Band technology, Wi-Fi, WiMax and Bluetooth the wireless can be achieved. In addition, widening the coverage area and long distance transmission are improved by FOS (Fibre Optic Sensors) [15]. Because of its light weight nature, it do not suffer electromagnetic interference [16]. As a result of its advantages like low cost, self-organization, high reliability and distributed activity, the use of WSN has gained lot of attention in the recent years along with in the coal mine location system it has become a hot research point [17]. In the extraction of WSN information the location service is important. Particularly, in the real time underground data about the location of miners, most of the sensory data with location information is important [18,19]. To understand various techniques in WSNs, many localization frameworks and algorithms are suggested to understand the exact localization [20]. WSN provide benefits such as operational simplicity, improved coverage, small size and low cost when compare to the traditional wired sensors [21]. This research examines the advantages and disadvantages of utilizing drones in the planning, construction, and control of intelligent urban areas. This study discusses the significance and benefits of utilizing UAVs for planning, constructing, and managing smart cities. Moreover, it provides an overview of the different types, applications, and challenges associated with UAVs. In addition, block chain solutions for tackling the mentioned issues in UAVs within smart research areas and provided suggestions for enhancing the security and privacy of UAVs in smart cities [22].

The study [23] demonstrates the integration of EV charging systems in the smart grids especially with the utilization of ML techniques for optimization. The efficient energy control is essential for grid stability for the increase in the adoption of EV. Various ML techniques is examined for enhancing the charging scheduling, energy distribution and load forecasting. The enhancement in the performance of grid with less energy costs and the impact in environment is the ultimate goal. Similarly, the study [24] introduces a ML technique for enhancing a secured WSN for tackling various attacks, which the conventional methods has not involved. Thus, the study discovers the ML methods for predicting and transferring the secured breaches in real time. The main aim is to enhance the flexibility of WSN in reducing the computational slide and fake alarm rates. Alternatively, the study [25] introduces a DNN for predicting the accurate energy as the renewable energy such as solar and wind are highly variant as prediction is crucial for the stability. Also, the study examines several DNN optimization methods for enhancing the forecasting accuracy and effectiveness in computing. The main goal is to improve the energy control and implementation of renewables to the power systems.

On a real time basis, the technology is accomplish of online monitoring of underground working environment and ordering the collected sensed data at a above ground of central station to avoid the possibility of accidents and ensure the health and safety workplace environment. Many existing research approached various algorithm in WSN to analyze the positions of workers in underground mine. But most of the research concentrated only on positioning or else the leakage of hazardous gas. To overcome this issue, the proposed research uses modified precise DV (Distance Vector)-hop localization algorithm to analyze the positions of the workers. Additionally, all nodes are connected by the anchor nodes by proposed DV-hop method. The proposed technique also shows the nodes which are away from the communication frequency of the anchor node, then it will send the alert message to the control room with the statement of rescue the workers, gas leakage. This shows the proposed model have high communication range.

### 1.1 Motivation of the study

The motivation of the proposed study is to improve the efficiency and consistency of WSN (Wireless Sensor Networks), specifically under complex circumstances such as underground mining and in order to prevent the gas leaks which present significant safety hazards, potentially causing explosions or toxic exposure. Maintaining temperature control is challenging due to variable underground conditions, which can lead to heat stress or equipment failure. Tracking workers in real time is difficult in such environments, complicating safety monitoring and emergency response along with the security related with the communication failures along with localization of node, then the proposed study aims to mitigate the calamities and enhance the efficiency. In addition to that proposed study pursues towards the development of advanced algorithms which can adapt to dynamic situations and ensures a dynamic data transmission. Hence, the motivation of the study is to contribute towards security with effectual monitoring systems, which can operate in opposing conditions. The study is dynamic for evolving technology under crucial systems where protection is dominant.

### 1.2 Research contribution

The primary objectives of the proposed research as follows:

• The data used in the proposed work is collected from the sensor nodes and segregate as an anchor nodes and wireless sensor nodes.
• To analyze the wide range of nodes from anchor nodes after parameter initialization for safety alert using proposed modified precise DV-hop node localization algorithm by extract the critical data.
• The efficiency of the proposed model is evaluated by using accuracy metric and calculate the distance between hop nodes precisely.

### 1.3 Paper organization

The following paper is allocated into four segments. Section II includes the existing model with different localization algorithm in WSN. Section III reflects the complete methodology of the entire study with their corresponding algorithms. Section IV includes the overall results and analysis of the proposed modified precise DV-hop node localization algorithm. Section V shows the conclusion, limitation and the future work of the proposed model.

## 2 Literature review

The existing research [26] implemented an intelligent system to improve the safety for coal mine employees. By utilizing the WSN the existing research has been collected the surrounding data such as groundwater level, earth pressure, harmful gases, humidity data and vibration. To minimize the delay between energy optimization and end nodes by location based energy efficient routing protocol. Likewise, the suggested research [27] demonstrated the prototype of mine safety system planning and construction. To determine WSN the existing research has been uses Zigbee technology. The WSN has been attained average performance. Literally, the considered research [28] implemented the system of smart safety monitoring with improved DV-Hop localization algorithm for appropriate positioning. It has been useful for analyze the casualty by send the early warning. The system has been attained average performance. Similarly, the prevailing research [29] demonstrated the localization algorithm to analyze the signal strength and distance. It has been based on Dual predict and RSSI (Received Signal Strength Indicator) algorithm to analyze the workers’ signal. The system has been attained better performance. Correspondingly, the existing research [30] implemented the RSSI based improved weighted centroid localization algorithm for underground coal mining area. Based on minimum RMSE (Root Mean Square Error) criteria, the exponential factor has been enhanced by improved quantum PSO (Particle Swarm Optimization). The system has been attained average performance. Likewise, the considered research [31] recommended improved entropy based RSSI localization algorithm has been used to analyze the positions of workers. The node location has been identified by the localization technique based on genetic algorithm. The model has been attained better performance. Literally, the suggested research [32] demonstrated the RSSI based positioning technique for analyze the signals of underground coal mine workers. In coal mines, the RSSI correct value has been predicted by weighted-entropy model. The model has been attained better performance. Similarly, the existing research [33] implemented the RIS (Reconfigurable Intelligent Surface) resource allocation and JCAS (Joint Communication and Sensing) to improvise the wireless surrounding. The RIS phase matrix optimization sub-problem has been shifted by based on the algorithm of SCA (Successive convex approximation). The system has been attained average performance. Correspondingly, the prevailing research [34] demonstrated the localization algorithm to find out the locations of the workers in coal mining area. The model gas been attained average performance. Likewise, the considered research [35] implemented the IoT based DSICS (Dynamic Sensor Information Control System) to analyze the dangerous carbon emissions, warm humidity and precipitation. The technique has been attained better performance.Beisdes, in the existing study [9], data is transmitted wirelessly using protocols like Zigbee or LoRa to a central processing unit, reducing wiring needs. Advanced algorithms analyze this data to assess conditions and predict hazards, enabling real-time alerts.

The prevailing research [36] recommended a smart IIoT (Industrial Internet of Things) in coal mine for safety monitoring of crowd sensing. The existing research has been used PSO Elman NN (Neural Network) and ADI-LSTM (Analog to Digital Converter Interface- Long Term Short Term Memory) for analyze the positions of human and supporting machines pressure values. The technique has been attained average performance. Literally, the considered research [37] demonstrated the network of smart phone for sensor data communication to the surface from the underground production environment by RSS (Received Signal Strength). The method has been attained better performance. Similarly, the suggested research [38] implemented the wireless data transmission technology and bus technology based coal mine monitoring signal transmission. The methods has been attained better performance. Correspondingly, the existing research [39] demonstrated the safety monitoring in coal mines based on WSN by lightweight AKA (Authentication and Key Agreement) scheme with AVISPA (Automated Validation of Internet Security Protocols and Applications) tool. To analyze the formal and informal security analysis by ROM (Random Oracle Model). The model has been attained average performance. Likewise, the prevailing research [40] implemented the RFID (Radio Frequency Identification) and adaptive heuristic mathematical model on IoT-based for monitoring the coal mining environment. The model has been attained better performance in verification of the miner's position, signal tracking and detection of suspicious incidents. Literally, the considered research [41] demonstrated routing algorithm namely SSAM (Sensory Swarm Autonomous Monitoring), reactive and proactive for extended sensor network. The method has been attained better performance. Likewise, the suggested research [42] implemented the positioning technique based RSS (Received Signal Strength) and RFID (Radio Frequency Identification) has been combined to detect the locations of mine's workers. The recommended model has been compared with WKNN (Weighted K-Nearest Neighbor) and the recommended model has been attained better performance. Similarly, the existing research [43] demonstrated the communication cost and residual energy-based C-EEUC (Centralized Non-Uniform Clustering) routing protocol and better performance has been attained by the approached method. Correspondingly, the existing research [44] demonstrated the model based on RF (Random Forest) underground location algorithm. In the real time and offline sampling stage the Kalman Filter algorithm has been analyzed the RSS. The method has been attained average performance in location accuracy. Literally, the prevailing research [45] implemented the hybrid sensor deployment approach of grid and multi-level methods in a linear and incorporated mine networks. The hybrid method has been attained better performance.

The considered research [46] approached IAUKF (Improved Adaptive Unscented Kalman Filter) has been used to resolve the transmission fault and signal fluctuation. The improved Sage – Husa noise estimation method has been used to analyze the unknown noises. To split the spatial distribution sensors into numerous clusters by multi-sensor clustering. Literally, the suggested research [47] implemented the hybrid approach of MEREC-CoCoSo (Method for Eliciting Relative Weights - Combined Compromise Solution). The MEREC has been used to determine the criteria weight, sensor and criteria discernment and the MEREC-CoCoSo has been used for sensor polarization. The model has been attained average performance. Likewise, the prevailing research [48] demonstrated the enhanced DEECP (Distributed Energy-Efficient Clustering Protocol). The recommended model has been compared with DEECP. The recommended model has been attained better performance. Similarly, the existing research [49] implemented the HWO (Harmonic Water Optimization) and HMP (Harmony Management Preprocessing) to make sure the water quality and preprocess the dismissed and uncertain data. The data quality has been improved by the HFC (Heuristic Fusion Clustering). The recommended model has been attained better performance. Correspondingly, the prevailing research [50] demonstrated the approach of efficient relay deployment for underground coal mining. The recommended research has been improved the lifetime coverage of parameter. Literally, the existing research [51] implemented the sensor based crack detection by using UHF (Ultra High Frequency), RFID (Radio Frequency Identification) in coal mining conveyor belts. A dielectric significance of the belt has been executed with aim of enabling the performance of conveyor belt sample. The better performance has been attained by the approached model. Likewise, the considered research [52] demonstrated the VLC (Visible Light Communication) has been integrated with SNR (Signal to Noise Ratio) has been approached for detect the location of miners. To transmit the mining information to the surface control room by LoRa (Long Range) technology has been used. The model has been attained better performance. Similarly, the prevailing research [53] demonstrated the hierarchical clustered WSN by LEACH+ (Low Energy Adaptive Clustering Hierarchy).

The MATLAB has been used for simulation.The approached LEACH + has been compared with LEACH. The approached model has been attained improved performance in scalability, network lifecycle and energy consumption. Correspondingly, the existing research [54] approached 3D LIDAR (Light Detection and Ranging) based underground localization method. The underground mine worker's location has been achieved by DWM (Distance Weight Map). The model has been attained better accuracy. Literally, the suggested research [55] demonstrated the mobile terminal intelligent system to monitor and detect the safety in coal mine environment. The approached detection system has been constructed by GIS technology. The performance of the approached system has been attained average performance.

The study has introduced an optimal scheme to minimalize the energy consumption in WSNs by using clustering algorithms and an energy-efficient routing protocol. It uses the K-means clustering algorithm for node grouping and LEACH for efficient data transmission. The results show significant reductions in energy consumption, extended network lifetime, and improved overall efficiency in WSN operations [56]. The study has implied about several deployment strategies and energy-efficient methods in WSNs, such as LEACH for clustering and DEEC for energy-efficient routing. It has examined the impact of node placement on network performance and energy consumption. The results has obtained that the optimized deployment strategies and energy-efficient protocols significantly enhance network lifetime, reduce energy consumption, and improve overall system performance [57]. The study has suggested a data aggregation algorithm to enhance the performance of the SPEED routing protocol in WSNs. The algorithm has reduced redundant data transmission and minimizes energy consumption while maintaining low latency. The results show improved throughput, reduced energy usage, and enhanced network efficiency, particularly in large-scale WSNs [58].The study has examined several ad-hoc routing protocols for WSNs, including AODV, DSR, and TORA. It compares their performance based on metrics like latency, energy consumption, and scalability. The outcomes highlight that AODV offers better scalability and energy efficiency, while DSR performs well in low-latency scenarios, with TORA showing advantages in highly dynamic networks [59].

### 2.1 Problem identification

• The existing method has not been able to track the movement and location of the workers in the coal mining area [35].
• The limitation of the suggested research has been, in various coal production circumstances the traditional learning model does not deliberate privacy production and data distribution. In addition, during the complex production processes, the existing techniques has been faced difficulty to meet out the requirements due to lack of parameter optimization [36].
• The considered research has to improve the scalability and reliability of WSN in mining environment [41].

## 3 Proposed methodology

Monitoring the underground coal mining environment is one of the most difficult task in coal mining industries. To address this issue, the proposed research uses the modified precise DV-hop node localization algorithm to monitor the workers even if they are in out of coverage from the sensors. Moreover, DV-hop anchor node is defined as a node in a wireless sensor network, which is utilized for localization. The nodes have a definite position and helps in identifying the locations of the further nodes through distribution of co-ordinates and its amount of hops that to be reached.The modifications to the DV-Hop algorithm aim to improve localization accuracy and communication range, especially in coal mine environments. Key changes include:

1. **Enhanced Anchor Node Selection**: Prioritizing stable and reliable anchor nodes to reduce localization errors.
2. **Distance Estimation Improvement**: Using advanced metrics like weighted distances based on signal strength or time of arrival for more precise distance estimates.
3. **Adaptive Communication Ranges**: Adjusting transmission power and frequency to adapt to environmental factors such as obstacles and interference in coal mines.
4. **Error Correction Techniques**: Implementing error correction to address issues like multipath propagation and signal fading, improving accuracy.
5. **Iterative Refinement Process**: Refining initial estimates through multiple rounds of communication to reduce inaccuracies over time.

These modifications collectively enhance the algorithm's ability to function effectively in challenging underground conditions. The complete flow of the proposed mechanism is depicted as Fig. 1.

**Fig. 1:** Mine safety monitoring system based on WSN [9].

Fig. 1 demonstrates that initially the dataset is created by the nodes and it will generate 2 categories of nodes such as anchor nodes and wireless sensor nodes. Moreover, the anchor nodes have some advantages such as providing reference points for localization that assist in increasing the accuracy of the non-anchor nodes positions. However, the localization accuracy is less if there is a limited number of nodes in the complex environment. Similarly, the sensor nodes have certain benefits, it assist in collecting data from nodes and it can be deployed in greater numbers for increasing the coverage area and it has limited power with processing capabilities, which interrupt the collection of data. It is considered as a drawback for the sensor nodes. Addition to that the gateway nodes are used to facilitate connection among the sensor nodes with the exterior network, which aggregates the data for effective transmission. If there is an overload there is an occurrence of bottleneck issues which leads to shorter operational time. Moreover, a relay nodes are used to extend the communication by relaying data and nodes, which improves the reliability of the network through adjacent paths and the introduction of latency under data transmission can require further energy resources. Moreover, the parameters such as network parameters, proposed localization algorithm parameters, simulation parameters and safety monitoring parameters are initialized. The wireless sensor network (WSN) in coal mine environments is defined by key parameters: Node density, which ranges from 5 to 20 nodes per 100 square meters, balancing accuracy and communication overhead; Communication range, typically 10–50 m, depending on terrain and conditions; and the Anchor node ratio, recommended at 20–30 % of total nodes, influencing localization accuracy. The localization algorithm parameters for the modified DV-Hop algorithm include Hop Count, which is measured during simulation and affects accuracy, with fewer hops leading to better results. Distance Estimation Error should ideally be less than 5 % of the actual distance to minimize impact on accuracy. Localization Accuracy aims for over 90 % accuracy, with nodes correctly localized within a defined threshold distance in optimal conditions. The safety monitoring parameters in coal mines include a temperature threshold of 60 °C, methane levels above 1.0 %, carbon monoxide above 50 ppm, and humidity levels between 30 % and 70 % relative humidity, all critical for ensuring safety in the mining environment.

Table .1 depicts the comparative results of the proposed Modified Precise DV-Hop with the traditional DV-hop in which the localization accuracy is increased to 92 % and the error value is decreased to 3 % in the proposed algorithm.

**Table 1:** Localization accuracy of modified Precise DV-hop.

Algorithm	Number of Nodes	Correctly Localized Nodes	Localization Accuracy (%)	Distance Estimation Error (%)
Traditional DV-Hop	100	75	75 %	8 %
Modified Precise DV-Hop	100	92	92 %	3 %

Then the proposed modified precise DV-hop node localization algorithm is utilized for collecting the sensor data collected by the nodes. The localization of the nodes are improves by MATLAB simulation. During the simulation the process extract the critical sensor data and analyze the safety data, the threshold value and alert mechanisms are added. The proposed model will also shows the nodes with are higher than the threshold value at that time it will trigger the alert mechanism. Through the simulation process the accuracy and efficiency of the proposed modified precise DV-hop node localization algorithm are evaluated by the performance metrics and it will finally improve the safety production.

### 3.1 Node formation

In underground mining areas, the most important role to make sure the effective data collection and reliable communication by node formation. Throughout the underground mining area, the node formation requires organizing WSN nodes to overcome the encounters such as signal reduction by launching specialized communication infrastructure. To facilitate effective data collection and communication these nodes are organized into topology such as hybrid, star and mesh. When the power management approaches improve the energy usage for extended node lifespan enable the localization algorithm to precise node tracking. To make sure the continuous network operation while the protocols adjust dynamically to altering the underground conditions by data routing and aggregation algorithms. Fig. 2 shows the node formations in WSN.

**Fig. 2:** Overall Process of Proposed model.

Fig. 2 shows the Node formation process in WSN. The figure shows two different nodes, the node with blue color are sensor nodes and the nodes with red color are anchor nodes. Each anchor nodes connected with two or more sensor nodes to pass the information. The information of the worker's positions are collected by these nodes and send the safety alert message to ground center in case of any emergency. Moreover, a buffer in the node acts as a short-term storage region for incoming and outgoing data. It assist in managing the flow of data, and conforming that the node has the capability to burst the traffic deprived of information loss. Besides, buffer can maintain smooth communication. During the storage of incoming data, the arrived data packets are stored in the buffer initially. The node process the packets in an order and ensures that no data is lost in the processing speed, which is less than incoming data rate. Similarly, in the outgoing data storage, the data packets are send formerly, where the node is placed in the buffer for managing the transmission process. It allows the node to highlight the packets based on insistence or significance, maximizing the communication efficacy. If the buffer is full, then data dropping is done. Where the earliest or minimum significant data packets are discarded and the space is created for the imminent incoming data, which is widely used in real-time systems. The flow is controlled by pausing the data transmission till the space is available for buffer and permitting the node to process the prevailing data.

### 3.2 Localization algorithm

#### 3.2.1 Traditional DV (Distance vector) - Hop localization algorithm

In accordance with the distance vector routing protocol, a distributed range free localization algorithm is DV-Hop localization. To evaluate the distance between unknown/unidentified and beacon nodes, multiple the AHD (Average Hop Distance) in WSNs using the hop count of the beacon nodes is used. Realizing the localization through multilateration, trilateration and triangulation the unknown nodes position information is attained. Furthermore, WSNs confronts different attacks which involves jamming, sinkhole attack and eavesdropping. For mitigating these threats, the resolution can be provided secured data transmission by encrypting the protocols. Whereas, the redundant routing techniques may improve resilience compared to node failure. In addition to that interruption detection systems aid in finding and respond to skeptical activities, also ensures integration of the network. By implementing these approaches, there is a significant enhancement in the security and reliability of WSNs. The 40 routes of beacon nodes from unidentified nodes are not probably narrow for a topology of network recognized by an unsystematic organization of WS nodes. The DV-Hop algorithm is mainly distributed into 3 stages. Firstly, it calculate the least hop count between the unknown nodes and beacon nodes. Through the protocol of classical distance vector routing that express their locations to nearby nodes by beacon nodes broadcast information. The information contains $\{\text{id},a_{i},b_{i},H_{i}\}$, here id $\left(a_{i},b_{i}\right)$, and the identifier is denoted by $H_{i}$. The i represent the beacon nodes hop count and the coordinate. For $H_{i}$ the initial value is set to zero. The transferring information are received by the nodes and record its localization and beacon nodes hop counts arc considered as vectors and then transmitted to neighbouring nodes. It is hypothetical to parallel $H_{i}$, the newly attained value once a node obtains the same id group with original value and to update and replace the original group by select the minimum value. By this communication node in WSNs, the minimum hop count and its position information of all beacon nodes are attained.

Secondly, to assess the distance between beacon and unidentified nodes by evaluating the minimum hop count and AHD. The average hop distance of complete network can be calculated after acquiring the hop count and localization of beacon nodes in the initial stage. To all network the information is broadcast. Where the AHD is denoted by $hd_{i}$ and h(ij), the beacon node is represented as $i\;\left(a_{i},b_{i}\right)$, the unknown node is signified as $j\;\left(a_{j},b_{j}\right)$. The formula shown below.

(1) $$hd_{i}=\frac{\sum \sqrt{{\left(a_{i}-a_{j}\right)}^{2}+{\left(b_{i}-b_{j}\right)}^{2}}}{\sum h\left(ij\right)}$$

By using the below formula the distance between unidentified and beacon nodes are estimated.

(2) $$d_{i}=hd_{i}\times Hop\text{,}$$

The AHD is represent by $hd_{i}$ the minimum hop count between the beacon nodes and unknown nodes are represent by Hop.

Finally, the $\left(a_{1},b_{1}\right),\left(a_{2},b_{2}\right)$ and $\left(a_{3},b_{3}\right)$ are BEACON1,BEACON2,BEACON3 the coordinates of three beacon nodes. The distance(a,b) denotes the distance between unidentified nodes and three beacon nodes and it is stated as $d_{1},d_{2},d_{3}$ distinctly. The formula obtained below.

(3) $$\left\{\begin{array}{c} \begin{array}{c} {\left(a_{1}-a\right)}^{2}+{\left(b_{1}-b\right)}^{2}=d_{1}^{2}\\ {\left(a_{2}-a\right)}^{2}+{\left(b_{2}-b\right)}^{2}=d_{2}^{2} \end{array}\\ {\left(a_{3}-a\right)}^{2}+{\left(b_{3}-b\right)}^{2}=d_{3}^{2} \end{array}\right\}$$

By the following formula the coordinate of node d is calculated.

(4) $$\left[\begin{array}{c} a\\ b \end{array}\right]={\left[\begin{array}{c} 2\left(a_{1}-a_{3}\right)\;2\left(b_{1}-b_{3}\right)\\ 2\left(a_{2}-a_{3}\right)\;2\left(b_{2}-b_{3}\right) \end{array}\;\right]}^{-1}*{\left[\begin{array}{c} \begin{array}{c} 2\left(a_{1}^{2}-a_{3}^{2}+b_{1}^{2}-b_{3}^{2}+d_{3}^{2}-d_{1}^{2}\right)\; \end{array}\\ 2\left(a_{1}^{2}-a_{3}^{2}+b_{2}^{2}-b_{3}^{2}+d_{3}^{2}-d_{2}^{2}\right) \end{array}\right]}^{-1}$$

(5) $$X={\left(A^{T}A\right)}^{-1}A^{T}b$$

The unknown nodes coordinates are calculated by this way. The routes from beacon to unidentified nodes are not probably narrow for a topology of network recognized using unsystematic arrangement of WS nodes. When using the traditional DV-Hop algorithm certain errors occur in the localization process. During, transmission if the neighbouring node is faulty, then it utilizes an alternate path and reaches the destination by bypassing the faulty node. Similarly, if the sender communicates with redundant nodes, then it can take the backup of the faulty node. By implementing the error detection and recovery mechanism, the faulty nodes are identified through triggering the recovery protocols.

#### 3.2.2 Proposed modified precise DV (Distance vector) - Hop localization algorithm

To overcome the issue in traditional DV-Hop algorithm, the proposed research use modified precise DV-Hop localization algorithm. Depending on an unbiased estimation, equation (5) shows the traditional way to fetch the average hop size. Based on the following equation the estimation method is optimized.

(6) $$Z_{1}=\left[\frac{1}{T-1}\sum_{j\neq i}{dis}_{ij}-HOPS_{j}^{D}*h_{ij}\right]$$

Here, the count of anchor nodes are denoted as T, The distance and hob count between i and j anchor nodes are denoted as ${dis}_{ij}$ and $h_{ij}$. The estimated average hop size is denoted as $HOPS_{j}^{D}$. To get the estimation of $HOPS_{j}^{D}$ by let the value of formula (5) to be zero. By this method, the mean value of estimated error attained zero. On the other hand, generally in some cases deviation or variance is more reasonable than MSE (Mean Square Error), if comprehending the error obey Gauss distribution. To calculate the hop size, the proposed research uses the minimum MSE criterion. It requires to minimize the formula value of equation (7) to get the average hop size $HOPS_{j}^{R}$.

(7) $$Z_{2}=\left[\frac{1}{T-1}\sum_{j\neq i}{\left({dis}_{ij}-HOPS_{j}^{R}*h_{ij}\right)}^{2}\right]$$

(8) $$let\frac{\partial g_{2}}{\partial HOPS_{i}^{R}}=0$$

The estimated average hop size can be attain:

(9) $$HOPS_{i}^{R}=\sum_{j\neq 1}\frac{h_{ij}{dis}_{ij}}{\sum_{j\neq 1}h_{ij}^{2}}$$

The size of average hop is projected by A and calculated as $\frac{\left(40+100\right)}{\left(2+5\right)}=20$ with the traditional method. Likewise, 24 and 22.5 would be the calculated B and C hop size. The proposed modified precise DV-Hop localization algorithm calculated the size of average hop is projected by A as $\frac{\left(40*2+100*5\right)}{\left(2*2+5*5\right)}=20$ and likewise, 24.6 and 21.76 would be the calculated B and C hop sizes. In a sensor network the distribution of anchor nodes are might not be identical. It is challenging to replicate the nodes distribution in the overall network, in case the average distance for every hop projected through a specific anchor node is utilized. In the calculation of positioning results, the large deviation is occurs with the space towards further anchor-nodes, if the unknown node utilizes the anchor node normal distance per hop. The multiple anchor nodes requires average distance per hop is deliberated to enhance the accurateness by computing the anchor nodes average distance for every hop. The explanation of its state of native network is dissimilar against the anchor nodes those hops are dissimilar for the same unidentified node. The dissemination of the unknown node native network is represent precisely by the anchor node which is nearer to the unidentified node. The unknown node hop value should be larger than the anchor node weight which is smaller. The projected anchor node average hop distance *i* is $P_{i}$, the number of unknown node hops between the anchor node *i* are denoted as $R_{i}$. The average hop distance weight can be estimated as follow in case the indefinite node gets a n anchor nodes data packets.

(10) $$V_{i}=\frac{\frac{1}{R_{i}}}{\sum_{j=1}^{n}\frac{1}{R_{j}}}$$

To all the anchor nodes, in equation (10) it shows that i anchor node is divided using the proportional addition of the unidentified node hop value and the anchor node i weight is equivalent to the ration of the hop value of the indefinite nodes. The weights sum of every anchor node is definite to be 1 through the method of normalized processing. In the positioning result, the greater weight value may minimize the deviation occurred by the remote anchor node and unknown node according to the modification in the hop value. To calculate the AHD of the unknown node, the corresponding formula can be used depend on the hop weighted DV-Hop algorithm.

(11) $$P=\sum_{i=1}^{n}V_{i}P_{i}$$

Hence, the anchor nodes are not project the AHD of the unknown nodes only some of improved algorithm utilizes. By the anchor nodes there is a great impact to the distance of average hop. A key problem is how to select the anchor nodes. To solve this problem, the proposed algorithm presents modified algorithm that is while computing the indefinite nodes AHD the anchor node will be skipped in case the number of hops among the unknown node and an anchor node is higher than the threshold, or else for estimating AHD for the unknown node by utilized the weighted method. The localization outcomes will be near to the closer nodes in entire anchor nodes by reduce the circle radius of the weight method. In certain cases, the projected unknown nodes are turned into anchor nodes if the indefinite nodes have no anchor nodes. equation (12) illustrated that the average error function is also defined as localization error.

(12) $$L_{error}=\sum_{i=m+1}^{R}\sqrt{\frac{{\left(A_{i}^{\prime }-A_{i}\right)}^{2}+{\left(B_{i}^{\prime }-B_{i}\right)}^{2}}{R*\left(R-T\right)}}$$

The real coordinates of unknown node i is represent as $\left(A_{i},B_{i}\right)$, the projected coordinate of the indefinite node represents as $\left(A_{i}^{\prime },B_{i}^{\prime }\right)$, the sensor nodes communication radius are denoted as R. Within the sensor field the entire number of nodes are represent as N. The amount of anchor nodes are represent as T. The below table shows the overall flow of process involved in the proposed algorithm.

Fig. 3 show the entire process of proposed modified precise DV-Hop localization algorithm. Initially, it collects the locations of anchor nodes and its hop counts and set up the initial average hop size. Here, the proposed modified precise DV-Hop localization algorithm is apply to calculate the Euclidean distance to define the distance between all pairs of anchor nodes and calculate the average hop size. Based on the distances between anchor nodes, the average hop size is estimated by MSE (Mean Square Error). If the value of MSE is less than threshold value it determine that MSE between the actual hop counts and the estimated hop counts exceeds the threshold. Proceed with the average hop size updation. To minimize the MSE adjust the average hop size and assign the location of unknown nodes. To evaluate the locations of unknown nodes by using the final average hop size. If there is a major increase in hop count during the examination then check for emergency conditions. If the emergency is detected as yes, then activate safety alerts because of emergency conditions and evaluate the safety parameters. Check the safety parameters such as temperature, gas leakage, air humidity and workers rescue and then complete the process. The component and simulation parameters of the proposed algorithm shown in Table 2.

**Fig. 3:** Node formation.

**Table 2:** Components of proposed algorithm.

Component	Description	Range/Value
Number of Anchor Nodes	Number of anchor nodes	5
Number of Sensor Nodes	Number of sensor nodes	20
Communication radius	Communication radius for sensor nodes	10
Anchor Nodes	Coordinates of anchor nodes	Uniform distribution in [0, 1] for both x and y coordinates (5, 2)
Sensor Nodes	Coordinates of sensor nodes	Uniform distribution in [0, 1] for both x and y coordinates (20, 2)
MP dv Hop Anchor Nodes	Modified DV-Hop sensor nodes' coordinates	Uniform distribution in [0, 1] for both x and y coordinates (5, 2)
MP dv Hop Sensor Nodes	Modified DV-Hop sensor nodes' coordinates	Uniform distribution in [0, 1] for both x and y coordinates (20, 2)
Dv Hop Anchor Node Assignments	Sensor nodes assigned to each anchor node	Computed in code
Nodes Per Anchor	Sensor nodes per anchor node	4 (approx.)
Num Extra Nodes	Number of extra nodes added	50
Dv Hop Extra Nodes	Extra nodes' coordinates	Uniform distribution in [0, 1] for both x and y coordinates (50, 2)
X	Loaded estimated coordinates	Estimated coordinates
Min Hop Count	Minimum hop count for connections	1, 2, 3
MP dv Hop Error Distances	Error distances for unknown nodes	$\sqrt{{\left({ux}_{i}-{ux^{\prime }}_{i}\right)}^{2}+{\left(uy_{i}-{uy^{\prime }}_{i}\right)}^{2}}$
Dv Hop Mean Error Distance	Mean error distance for localization	$\frac{1}{N_{i}}\sum_{i-1}^{N_{u}}\sqrt{{\left({ux}_{i}-{{ux}^{\prime }}_{i}\right)}^{2}+{\left({uy}_{i}^{i}-{uy^{\prime }}_{i}\right)}^{2}}$
Threshold	Error distance threshold	0.2 (The error distance threshold is a user-defined parameter that determines the acceptable level of error for localization)
Safe Nodes	Nodes with error distance≤threshold	The count of unknown nodes with an error distance less than or equal to the specified threshold.
Emergency Nodes	Nodes with error distance > threshold	The count of unknown nodes with an error distance greater than the specified threshold.
Avg Anchor Distance	Average distance between anchor nodes	$\frac{1}{\frac{N_{a}\left(N_{a}-1\right)}{2}}\sum_{i-2}^{N_{a}}\sum_{j-i+2}^{N_{a}}\sqrt{{\left({ax}_{i}-{ax^{\prime }}_{j}\right)}^{2}+{\left({ay}_{i}-{ay^{\prime }}_{j}\right)}^{2}}$
Avg Anchor Sensor Distance	Average distance between anchor nodes and sensor nodes	$\frac{1}{\frac{N_{a}\left(N_{u}\right)}{1}}\sum_{i=2}^{N_{a}}\sum_{j=1}^{N_{u}}\sqrt{{\left({ax}_{i}-{ux^{\prime }}_{j}\right)}^{2}+{\left({ay}_{i}-{uy^{\prime }}_{j}\right)}^{2}}$
Scaling Factor	Computed scaling factor	Scalingfactor= $\frac{Average\;distance\;between\;anchor\;nodes}{Average\;distance\;between\;anchor\;nodes\;and\;sensor\;nodes}$
total_nodes	Total number of nodes (for plotting)	50
proposed_dv_error	Average localization error for plotting	The average Euclidean distance between the actual position and the estimated position of all the unknown nodes.

### 3.3 Safety parameters initialization

#### 3.3.1 Analyses of critical parameters

The total energy need for retrieval and storage of events in WSNs are maximum as the some values in parameters of WSNs increase. Table 2 shows the critical parameters of WSN.

**Table:** 

**Parameters of WSN**
**1.**Fromthesinkcalculatethedistanceofsensornodes **2.**$\left(|{\text{Path}}_{i,sink}|,\text{for}\;\text{sensor}\;\text{node}\;i\right)$ **3.**Calculatethequantityofdatatransferredtobeaconnodesthroughsensornode **4.**Calculatethequantityofdatatransferredtothesinkthroughbeaconnodes **5.**$\text{From}\;\text{beacon}\;\text{nodes}\;\text{calculate}\;\text{the}\;\text{sensor}\;\text{nodes}\;\text{distance}\;\left({\text{Path}}_{i,j},\text{for}\;\text{sensor}\;\text{node}\;i\;\text{and}\;\text{beacon}\;\text{node}\;j\right)$ **6.**$\text{From}\;\text{the}\;\text{sink}\;\text{calculate}\;\text{the}\;\text{beacon}\;\text{nodes}\;\text{distance}\;\left({\text{Path}}_{j,\text{sink}},\text{for}\;\text{sensor}\;\text{donor}\;j\right)$ **7.**Frombeaconnodesmemorynumbercalculatethequantityofdatawrittentoorread

The characteristics of energy requirement for event retrieval and storage in WSN are provided by the critical parameters of Table 3. To identify the dominant critical parameters aid to increase the usage of available memory and minimize the cost of event retrieval and storage in WSN. The critical parameters shown in Table 4.

**Table 3:** Critical parameter.

Component	Description	Range/Value
temperature	Temperature for emergency nodes	Values between 20 and 40 °C
gas Leakage	Gas leakage indicator for emergency nodes	Values of 0 (no leakage) or 1 (leakage)
air Humidity	Air humidity for emergency nodes	Values between 30 % and 80 %

**Table 4:** Safety alert message by nodes.

Node Number	Temperature	Gas Leakage	Humidity	Alert Message
Node 7	23 °C	1	62 %	• Check for gas leakage
				• Rescue the workers
Node 11	24 °C	0	38 %	• Check for abnormal air humidity
				• Rescue the workers
Node 12	23 °C	0	78 %	• Check for abnormal air humidity
				• Rescue the workers
Node 13	20 °C	1	31 %	• Check for gas leakage
				• Check for abnormal air humidity
				• Rescue the workers
Node 16	40 °C	0	56 %	• Rescue the workers

The proposed model analysis every nodes in the coal mining area by it anchor nodes. The alert messages are given by these three parameters mentioned in Table 4. The error distance between the unknown nodes in proposed modified precise DV-Hop localization algorithm is shown in Fig. 4.

**Fig. 4:** Process of proposed modified precise DV-Hop localization algorithm.

Fig. 4 shows the number of nodes detected within the threshold value 0.2 and outside of the threshold value. Here, the nodes 1, 2, 3, 4, 5, 6, 8, 9, 10, 14, 15, 17, 18, 19, 20 are detected within the threshold value. The other nodes such as node 7, 11, 12, 13, 16 are detected in outside of the threshold value. If the nodes are detected in unsafe zone then it will send a safety alert message to the control to take initial actions. Table 4 shows how the nodes gives alert to the control room in case of any emergency to avoid the disaster.

Table 4 shows the list of alert message send to the control room for node 7, 11, 12, 13 and 16. Because these nodes are detected in outside of the threshold value.

Table .5 depicts the Safety monitoring alerts of the Proposed Modified Precise DV-Hop in which the proposed algorithm has obtained lower temperature of 2, gas leak methane of 1 and humidity level of 1 when compared to the traditional algorithms.

**Table 5:** Safety monitoring alerts of the Proposed Modified Precise DV-Hop.

Condition	Traditional DV-Hop Alerts Triggered	Modified Precise DV-Hop Alerts Triggered
High Temperature (>60 °C)	5	2
Gas Leak (Methane >1.0 %)	4	1
Humidity Level (Outside 30%–70 %)	3	1

## 4 Result and discussion

This section shows the simulation outcomes of proposed modified precise DV-Hop localization algorithm. The simulation includes the comparison of traditional localization algorithm with proposed localization algorithm, estimated distance of sensor nodes and anchor nodes and it hop counts.

### 4.1 Simulation outcomes

Fig. 5 shows the error waveform plot for proposed modified precise DV-Hop localization algorithm. Proposed model can detect sensor nodes both within safe zone as well as outside safe zone of the region. The shows the proposed model has high communication range than compare to existing model.

**Fig. 5:** Error waveform for unknown nodes.

Table .6 depicts the communication range of the proposed Modified Precise DV-Hop in which the average communication range is increased to 40, maximum communication range is enhanced to 50 comparing to traditional algorithms.

**Table 6:** Communication range of the Proposed Modified Precise DV-Hop.

Algorithm	Average Communication Range (m)	Maximum Communication Range (m)	Node Density (nodes/100 m^2^)
Traditional DV-Hop	25	35	10
Modified Precise DV-Hop	40	50	10

Fig. 6 display the localization error of proposed algorithm. The figure shows the localization error attain by the traditional DV-Hop, proposed modified precise DV-Hop localization algorithm, Hop 1, Hop 2, Hop 3.

**Fig. 6:** Error Waveform for unknown nodes.

Fig. 7 shows the WSN with anchor nodes and estimated positions of traditional DV-Hop localization algorithm. The anchor nodes are connected with two or more sensor and it error distance are calculated by the estimation positions.

**Fig. 7:** Localization error of proposed algorithm.

Fig. 8 shows the minimum hop count 1 of proposed algorithm. Fig. 9 shows that the 1 hop count between one anchor node and one sensor node.

**Fig. 8:** Proposed method estimated positions of anchor nodes and WSN.

**Fig. 9:** Min hop count 1.

Fig. 9 shows the minimum hop count 2 of proposed algorithm. The figure shows that the 1 hop count between one anchor node and two sensor node. So the one count is nearer to the anchor node and the third count is little bit farer to the both anchor node and sensor node.

Fig. 10, Fig. 11 shows the minimum hop count 3 of proposed algorithm. The figure shows that the 1 hop count between one anchor node and three sensor node. So the one count is nearer to the anchor node, the second count is little bit farer to the both anchor node and sensor node and the third count is farer when compare to the first two sensor nodes (see Fig. 11).

**Fig. 10:** Min hop count 2.

**Fig. 11:** Min hop count 3.

#### 4.1.1 Comparative analysis

In this section the results of the proposed study is compared with the existing models and it is exposed in the detail.

With Attack.

Table .7 and Fig. 12, Fig. 13, Fig. 14, Fig. 15 depicts the performance metrics of different algorithms show notable variations in their efficiency. The K-Nearest Neighbors (KNN) algorithm demonstrated strong predictive abilities with a precision of 98.8 %, a recall of 98.1 %, and an F1 score of 98.5 %. The precision of Random Forest was 98.7 %, with a recall of 97.8 % and an F1 score of 98.3 %. On the other hand, the Naive Bayes classifier showed significantly worse results, achieving a precision of just 64.5 %, a recall of 54.9 %, and an F1 score of 59.1 %. The Decision Tree algorithm excelled, achieving a precision of 97.9 %, recall of 97.8 %, and an F1 score of 97.8 %. The algorithm proposed demonstrated superior performance compared to other models with exceptional metrics, achieving a precision and recall of 99.5 % each, along with an F1 score of 99.5 %, highlighting its accuracy in data classification.

**Table 7:** Comparison of proposed model with existing algorithms during attack.

Algorithm	Precision	Recall	F1 Score
KNN	98.8	98.1	98.5
Random Forest	98.7	97.8	98.3
Navie Bayes	64.5	54.9	59.1
Decision tree	97.9	97.8	97.8
Proposed	99.5	99.5	99.5

**Fig. 12:** Performance metrics of proposed model with existing algorithms during attack.

**Fig. 13:** Performance metrics of proposed model with existing algorithms - without attack.

**Fig. 14:** Performance metrics of proposed model with prevailing models [60].

**Fig. 15:** Performance metrics of proposed model with prevailing algorithms [60].

#### 4.1.2 Without Attack

Table .8 and Fig. 15 depicts the comparison of different algorithms emphasizes their varying levels of effectiveness in classification duties. The effectiveness of the K-Nearest Neighbors (KNN) algorithm was demonstrated by achieving impressive results: 99.2 % precision, 98.8 % recall, and an F1 score of 99, accurately identifying relevant instances. The Random Forest algorithm came in a close second, achieving a precision of 99 % and a recall of 98.3 %, leading to an F1 score of 98.7 %. Contrastingly, the Naive Bayes classifier showed notably inferior results, with a precision of 64.4 %, recall of 54.8 %, and an F1 score of 59.2 %. The Decision Tree algorithm also did very well, with a precision of 98.6 %, recall of 98.4 %, and an F1 score of 98.5 %. Nonetheless, the suggested algorithm excelled above the rest in terms of performance metrics, with a flawless precision and recall rate of 99.9 % and an F1 score matching this percentage, highlighting its remarkable classification abilities in comparison to the other models assessed.

**Table 8:** Comparison of proposed model with existing algorithms - without attack.

Algorithm	Precision	Recall	F1 Score
KNN	99.2	98.8	99
Random Forest	99	98.3	98.7
Navie Bayes	64.4	54.8	59.2
Decision tree	98.6	98.4	98.5
Proposed	99.9	99.9	99.9

In Table .9, Various models were assessed and shown to exhibit different levels of precision and recall measurements. The precision rate of the 2BSM model was 98.1 % with a recall rate of 98.5 %, showcasing strong performance. After analyzing the 2BSM model without taking into account attack scenarios, the results indicated a minor improvement, with a precision rate of 98.8 % and a recall rate of 99 %. However, the model showcased in the current study showed significantly reduced effectiveness, with 88.9 % accuracy and just 61.6 % recognition, indicating limitations in its capacity to accurately pinpoint pertinent instances. However, the proposed model stands out for its outstanding performance metrics, with a precision and recall rate of 99.5 %. This showcases its superior capability to precisely detect events compared to the other models assessed, indicating its potential for enhanced efficiency in practical situations.

**Table 9:** Comparison of proposed model with prevailing models [60].

Algorithm	Precision	Recall
2BSM model	98.1	98.5
2BSM model Without attack	98.8	99
Existing paper	88.9	61.6
Proposed	99.5	99.5

In Table 10, when comparing various algorithms based on F1 score and accuracy, noticeable variations in their performance are evident. The K-Nearest Neighbors (KNN) algorithm initially had a low F1 score of 78.8 % and accuracy of 86.3 %, but later achieved moderate scores of 86.6 % for F1 and 91.2 % for accuracy. The F1 score reached its highest point at 87.8 %, in addition to a notable accuracy rate of 91.6 %. In both the low and medium categories, the Random Forest algorithm demonstrated superior performance, with F1 scores of 84.7 % and 87.7 %, and accuracies of 90.6 % and 92.8 %, respectively. Nonetheless, its high-category performance saw a slight decrease, achieving an F1 score of 88.1 % and an accuracy of 92.7 %. The Stacking model exhibited similar trends, with F1 scores of 83.9 %, 86.6 %, and 86.7 % for low, medium, and high categories, while maintaining accuracies ranging from 90.2 % to 91.7 %. The proposed model excelled in every aspect, achieving perfect metrics with a low F1 score of 99.5 %, low accuracy of 99.3 %, and medium F1 and accuracy both at 99.5 %, while also preserving outstanding scores in the high categories. This demonstrates how the proposed model's superior performance in classification tasks surpasses the other algorithms evaluated.

**Table 10:** Comparison of performance metrics of proposed model with prevailing algorithms [60].

Algorithm	Low F1 Score	Low Accuracy	Medium F1 Score	Medium Accuracy	High F1 Score	High Accuracy
KNN	78.8	86.3	86.6	91.2	87.8	91.6
Random Forest	84.7	90.6	87.7	92.8	88.1	92.7
Stacking	83.9	90.2	86.6	91.5	86.7	91.7
Proposed	99.5	99.3	99.5	99.5	99.5	99.5

## 5 Discussion

In the discussion section the proposed model is compared with the various methods and it is depicted in Table 11.

**Table 11:** Comparison between different Methods with Proposed Model.

Ref	Model	Methodology Involved	Outcome Obtained	Proposed Work Results
[61]	QPSO algorithm	The weighted centroid formula is used by the algorithm to determine the coordinates, merging the intersection points of beacon nodes with their weights from RSSI measurements.	The improved algorithm showed a noticeably low mean square error (MSE) value of 0.330, demonstrating high precision in localization tasks.	The modified localization algorithm often integrates sophisticated methods like filtering and error correction, resulting in enhanced accuracy in positioning miners and equipment in comparison to the weighted centroid method, which may not address environmental factors as well.
[62]	Particle Swarm Optimization-Elman Neural Network (PE) algorithm	An algorithm named Particle Swarm Optimization-Elman Neural Network (PE) developed to predict the mobile human position. Furthermore, ADI-LSTM neural network forecasting model is used for predicting pressure readings of equipment foundations in underground mines.	PE algorithm demonstrates the smallest average cumulative prediction error and shows an increase in trajectory fit rate by 24.1 %, 13.9 %, and 8.7 % when contrasted with Kalman filtering, Elman, and Kalman plus Elman algorithms.	Research has demonstrated that the updated localization algorithm results in decreased average localization errors (e.g., 4.85 m) in comparison to conventional methods commonly utilized in crowd sensing applications, which typically lack precision.
[63]	PSO-BP model	The Levenberg-Marquardt algorithm was utilized for training, aiming to minimize the mean squared error (MSE) by adjusting the weights to match predicted and true outputs. Moreover, PSO algorithm mimics natural social behaviour patterns to optimize the initial weights of the BP neural network.	The MSE value of 2.0 × 10 ^−4^ attained by the improved PSO-BP model shows accurate predictions.	The modified localization algorithm in the WSN allows for immediate monitoring of miners and equipment, which is vital during emergencies. However, the PSO-BP neural network focuses on assessment and prediction rather than providing immediate location data for quick responses to hazardous scenarios.
[64]	Hybrid CNN-LSTM Architecture	The model utilizes CNN and LSTM networks to take advantage of their abilities in handling spatial and temporal data. CNN is employed to extract features from spatial data like images or environmental sensor data, whereas LSTM is used to understand temporal relationships in sequential data, which makes it appropriate for forecasting time-series data.	MHQI and concentration of CH4 gas, respectively. The mean RMSE values stood at 0.0322, 0.0320, and 0.0311 for MHQI, and 0.0230, 0.0222, and 0.0197 for CH4 gas concentration when employing CNN, LSTM, and a hybrid CNN-LSTM model.	WSNs enable real-time alerts by continuously monitoring environmental conditions such as gas levels and temperature using specialized sensors. The effectiveness of the CNN-LSTM model depends on analysing data derived from past trends, which might not be able to accurately detect abrupt real-time shifts.

Different algorithms for monitoring safety in coal mines are compared, showing different approaches and results. The QPSO algorithm achieves high localization precision with a low mean square error (MSE) of 0.330 using a weighted centroid formula based on RSSI measurements. On the other hand, the PE algorithm, combining Particle Swarm Optimization with Elman Neural Network, shows better trajectory fitting performance, resulting in a reduction of prediction errors by up to 24.1 % when compared to conventional methods. Additionally, the modified localization algorithm achieves an average localization error of 4.85 m. The PSO-BP model, using the Levenberg-Marquardt algorithm for weight adjustment, achieves an MSE of 2.0 × 10−4, demonstrating accurate prediction but without essential real-time localization for emergencies. Finally, the Hybrid CNN-LSTM structure integrates CNN for extracting features and LSTM (Long Short Term Memory) for handling temporal data, resulting in RMSE values of approximately 0.0311 for predicting gas concentrations. Yet, this model depends on past data trends, which might not accurately reflect abrupt shifts in the environment. In general, the updated localization algorithm in WSNs offers better accuracy and quick response abilities when compared to other methods, making it well-suited for the changing and risky environments found in underground coal mining.

The proposed solution addresses key challenges in coal mines, including real-time environmental surveillance for conditions like gas levels and temperature, worker and equipment localization for safety, and automated emergency alerts for rapid response. However, challenges such as communication disruption from dust and obstacles, sensor performance affected by environmental conditions, and complex node placement in mine layouts must be overcome. Additionally, handling high data volumes, ensuring low-latency processing, and addressing issues like scalability and node failure are critical for maintaining system reliability and effectiveness in real-world coal mine operations.

## 6 Conclusion and future recommendation

In coal mining industries, one of the main challenges has been formation of node in underground mining areas. Due to this structure, the mine workers has not been able to contact the ground staff in case of any emergency.In coal mines, gas leaks present significant safety dangers, possibly initiating explosions or toxic exposure. Retaining temperature control is challenging due to variable underground conditions, which can lead to heat stress or equipment failure. Tracking workers in real time is difficult in such environments, complicating safety monitoring and emergency response.To address this issue, and the proposed modified precise DV-Hop localization algorithm has been used to detect the movements of the workers in the coal mining area using WSN. The WSN has been suitable for these harsh environment because of its features such as multi-hop, flexible structure, self-organization, etc. The data has been collected from the generated nodes. The nodes has been formed as anchor nodes and sensor nodes. The network parameters, proposed localization algorithm parameters, simulation parameters, safety monitoring parameters has been included to analyze the environment and finally the proposed modified precise DV-Hop localization algorithm. The proposed algorithm has been compared with the traditional localization algorithm and the proposed algorithm has been attained high performance accuracy in sensor analysis than compare to traditional model. The proposed research has been used MATLAB to enhance the localization. The efficiency of the proposed model has been evaluated by simulations. However, the proposed study has certain limitations in scalability, accuracy, environmental factors, and energy consumption and with fault tolerance. The future work of the proposed research is planned to explore the effect of different patterns of node distribution on the performance of system.

## CRediT authorship contribution statement

**Hafiz Zameer ul Hassan:** Writing – original draft, Visualization, Validation, Investigation. **Anyi Wang:** Validation, Supervision, Project administration, Data curation, Conceptualization. **Ghulam Mohi-ud-din:** Writing – original draft, Funding acquisition, Conceptualization.

## Declaration of competing interest

The authors declare that they have no known competing financial interests or personal relationships that could have appeared to influence the work reported in this paper.

## Figures and Tables

**Table:** 

DV	Distance Vector
WSN	Wireless sensor network
AHD	Average Hop Distance
RSSI	Received Signal Strength Indicator
MSE	Root Mean Square Error
RSS	Received Signal Strength
LSTM	Long Short Term Memory
MATLAB	Matrix Laboratory
CNN	Convolutional Neural Networks
FOS	Fiber Optic Sensors
UAV	Unmanned Aerial Vehicle
KNN	K-Nearest Neighbors
PSO	Particle Swarm Optimization
QPSO	Quantum based PSO
